# Modulation of Vascular Smooth Muscle Cell Multiplication, Apoptosis, and Inflammatory Damage by miR-21 in Coronary Heart Disease

This article has been retracted.

**DOI:** 10.1155/2021/6942699

**Published:** 2021-11-27

**Authors:** Wei Liu, Yilin Li, Dongming Zhao

**Affiliations:** Health Care Clinic, Qingdao Municipal Hospital (Group), Qingdao, Shandong 266071, China

## Abstract

This study is aimed at exploring the role and potential molecular mechanism of microRNA-21 (miR-21) in coronary heart disease (CHD). RT-qPCR analysis was conducted to detect the expression of miR-21, Sprouty 1 (SPRY1), and connexin 43 (CX43). The protein expression of SPRY1 and CX43 was measured by western blot. ELISA was performed for measuring inflammatory factors, including intercellular adhesion molecule-1 (ICAM-1) and interleukin-1 beta (IL-1*β*). The target relationship between miR-21 and SPRY1 was determined by dual-luciferase reporter assay. Cell multiplication and apoptosis were detected using CCK-8 assay and flow cytometry analysis, respectively. Our results indicated that miR-21, CX43, and the level of inflammatory cytokines including ICAM-1 and IL-1*β* were upregulated, while SPRY1 was downregulated in blood samples from CHD patients compared with the controls. Besides, miR-21 directly targeted SRPY-1. miR-21 could suppress SPRY1 expression and enhance CX43 expression in VSMCs. Moreover, miR-21 accelerated cell multiplication and attenuated cell apoptosis in VSMCs. Collectively, these findings suggested that miR-21 could effectively elevate VSMC multiplication and repress apoptosis by targeting SPRY1 in CHD, providing a potential target for therapeutic strategy of CHD.

## 1. Introduction

Coronary heart disease (CHD) is a common cardiovascular disease usually resulted from atherosclerosis and has high mortality rate [1, 2]. There are multiple pathogenic factors of CHD, such as vascular stenosis, occlusion, myocardial ischemia, hypoxia, necrosis, inflammation, and cardiomyocyte apoptosis [3]. It has been reported that asthma, chronic obstructive pulmonary disease, or obesity will aggravate the disease of patients with CHD [4–7]. At present, the main treatment of CHD is cardiovascular interventional technique [8]. Although the treatment technology of CHD has made great progress, the prognosis of CHD patients is still worse due to the presence of comorbidities and the complexity of disease conditions [9, 10]. Accumulating evidence revealed that the aberrant proliferation of vascular smooth muscle cells (VSMCs) is a vital event in cardiovascular disease progression, including CHD [11, 12]. Moreover, inflammation and apoptosis are also major causes of the initiation and progression of CHD, which have been regarded as the prognosis indicators for CHD patients after treatment [13, 14]. Hence, it is of significance to explore the action of miR-21 on VSMCs in CHD progression.

MicroRNAs (miRNAs), a class of small noncoding RNAs (ncRNAs) with 22 nucleotides, could modulate the expression of target genes via binding to the 3′untranslated region (3′UTR) of mRNAs [15, 16]. In recent years, miRNAs were reported to participate in the progression of various diseases, including CHD [17, 18]. Previous studies demonstrated that miRNAs played vital roles in various biological functions, such as cell differentiation, proliferation and apoptosis in various diseases [19]. Of note, miR-21 was proved to exert important effects on the development of multiple human diseases. For example, miR-21 was elevated and exhibited the oncogenic effects on non-small-cell lung cancer development [20]. Moreover, absence of miR-21 enhanced cell apoptosis, vascular inflammation, and plaque necrosis during atherogenesis in macrophage [21]. It was reported that miR-21 was elevated in cardiovascular system [22]. A previous study indicated that miR-21 was associated with the risk and prognosis of CHD patients [23]. However, the role and underlying mechanism of miR-21 need further investigation. In the current research, the differentially expressed miR-21 in blood from CHD patients and VSMCs was analyzed. Furthermore, the action of miR-21 on inflammation response, VSMC proliferation, and apoptosis was explored in CHD.

## 2. Materials and Methods

### 2.1. Clinical Samples

The blood samples were obtained from 28 healthy volunteers (16 males and 12 females, age 35-74 years) and 30 patients diagnosed with CHD (19 males and 11 females, age 38-76 years) at the Qingdao Municipal Hospital from March 2020 to March 2021. 5 mL venous blood was collected from every participant and stored at -80°C.

Patient inclusion criteria are as follows: (1) patients met all the diagnostic criteria of CHD [24]; (2) patients were consistent with all the clinical symptoms of CHD and the characteristics of echocardiography combined with laboratory examination. Exclusion criteria are as follows: (1) women during childbirth or lactation, (2) serious impairment of liver and kidney function, (3) other coronary artery lesions, (4) other malignant tumors, and (5) other acute/chronic inflammatory diseases and/or autoimmune diseases that may impact the research.

This study was ratified by the Ethics Committee of the Qingdao Municipal Hospital, and all the enrolled participants and their families were informed and signed the informed consent form.

### 2.2. Cell Culture and Transfection

Human VSMCs (T/G HA-VSMC) purchased from Procell Life Science & Technology (Wuhan, China) were cultured in Ham's F-12K (Procell Life Science & Technology) with 10% FBS, 100 *μ*g/mL streptomycin, and 100 U/mL penicillin in an incubator containing 5% CO_2_ at 37°C.

For cell transfection, cells were inoculated into poly-D-lysine-coated 6-well plates at the concentration of 2 × 10^5^. Then, the sequences of miR-21 and the negative control (miR-NC) designed by Sangon Biotech (Shanghai, China) were transfected into T/G HA-VSMC cells using Lipofectamine 3000 (Thermo Fisher Scientific, Waltham, MA, USA).

### 2.3. RT-qPCR Analysis

Total RNA was extracted from the plasma or cells using TRIzol reagent (Yuanye Biotech, Shanghai, China). Total RNA purity was measured by ultraviolet spectrophotometer, and reverse transcription was conducted to synthesize cDNA using the PrimeScript™ RT Master Mix (Solarbio, Beijing, China). Then, qPCR was performed on the ABI7500 fluorescence quantitative PCR instrument (Long Jump Biological Science and Technology, Beijing, China) with the following qPCR cycling program: predenaturation at 95°C for 5 min, denaturation at 95°C for 15 s, and annealing and extension at 60°C for 30 s, for 40 cycles. U6 was used as the internal reference gene for detecting miR-21, and *β*-actin acted as the normalization for SPRY1 and CX43 mRNA expression detection. The expression of the relative genes was calculated using the 2^-*ΔΔ*Ct^ method. The specific sequences of the relative genes are listed in Table 1.

### 2.4. Western Blot

The proteins were isolated using RIPA lysis buffer (Beyotime, Shanghai, China). Protein concentration was determined by BCA protein determination kit (Thermo Fisher Scientific).The proteins were separated by 10% SDS-PAGE and then transferred onto a PVDF membrane (Millipore, Billerica, MA, USA). After blocking with 5% skimmed milk for 1 h, the membranes were incubated with the specific primary antibodies against SPRY1 (1 : 1,000, ab111523, Abcam, Cambridge, UK), CX43 (1 : 1,000, #3512, Cell Signaling Technology, Danvers, MA, USA), and *β*-actin (1 : 1,000, ab8226, Abcam) at 4°C overnight and the horseradish peroxidase-labeled goat anti-rabbit secondary antibody (1 : 5,000, ab6721, Abcam) for1 h at room temperature. Then, the protein bands were obtained using the ECL kit (Millipore). The gray value of the protein bands was analyzed using the Quantity One software.

### 2.5. Cell Multiplication Detection

T/G HA-VSMC cells were seeded into the 96-well plates. After transfection, 10 *μ*L CCK-8 solution (Beyotime) was added and cultured for 2 h. Finally, OD value (450 nm) was measured using a microplate reader.

### 2.6. Apoptosis Detection

To detect the number of the apoptotic cells, the transfected VSMCs were cultured in the 12-well plates. Then, the collected cells were washed using ice-cold PBS. Subsequently, cell suspension (1 × 10^6^ cells) was stained with Annexin V-FITC (RiboBio, Guangzhou, China) and PI (RiboBio) for 5 min without light. Finally, cell apoptosis of VSMCs was detected using flow cytometry (Beckman Coulter, Miami, FL, USA).

### 2.7. Measurement of Inflammatory Factors

Levels of inflammatory factors including intercellular adhesion molecule-1 (ICAM-1) and interleukin-1*β* (IL-1*β*) were determined by the corresponding ELISA kits.

### 2.8. Dual-Luciferase Reporter Assay

The connection between miR-21 and SPRY1 was predicted by TargetScan7.2 (http://www.targetscan.org/vert_72/). To form the SPRY1-Wt luciferase reporter vector, the wild-type (Wt) sequence of SPRY1 with the binding sites of miR-21 was cloned into the pGL3 vector (Promega, Madison, WI, USA). The mutated sequence of SPRY1 was used to construct the mutant (Mut) vector (SPRY1-Mut). T/G HA-VSMC cells were grown in the 96-well plates and cotransfected with miR-21 mimic and miR-NC, as well as SPRY1-Wt and SPRY1-Mut by Lipofectamine 3000 (Thermo Fisher Scientific). The firefly and ranilla luciferase activities were analyzed by dual-luciferase reporter assay (Promega).

### 2.9. Statistical Analysis

Data in this study were statistically processed by SPSS24.0 SPSS 19.0 (Asia Analytics Formerly SPSS China) and visualized via GraphPad Prism 7. The quantitative data were presented as the mean ± standard deviation (SD) and analyzed using Student's *t*-test. Correlation analysis was performed using Pearson's correlation coefficient. *P* < 0.05 was considered as statistically significant.

## 3. Results

### 3.1. Plasma miR-21, CX43, and SPRY1 in CHD Patients and Volunteers

The expression of miR-21 (Figure 1(a)) and CX43 (Figure 1(c)) was notably elevated, while SPRY1 (Figure 1(b)) was noticeably decreased in plasma from CHD patients in comparison to the controls. In terms of protein expression, CX43 was remarkably higher (Figure 1(e)), while SPRY1 (Figure 1(d)) was obviously lower in plasma from CHD patients than that in volunteers. The data identified an inverse connection between miR-21 and SPRY1 and between CX43 and SPRY1.

### 3.2. The Levels of ICAM-1 and IL-1*β* Were Elevated in CHD Patients

Comparing the contents of inflammatory factors in plasma from CHD patients and volunteers, we found that ICAM-1 and IL-1*β* were dramatically enhanced in CHD patients (Figures 2(a) and 2(b)). The correlation analysis revealed the positive association between miR-21 and ICAM-1 or IL-1*β*, suggesting that miR-21 induced the aggravation of inflammatory reaction (Figures 2(c) and 2(d)). These results revealed that inflammation response might be involved in the progression of CHD.

### 3.3. SPRY1 Was a Direct Target of miR-21

We predicted the potential binding sites between miR-21 and SPRY1 through TargetScan7.2 (Figure 3(a)). Dual-luciferase reporter assay showed that miR-21 mimic decreased the luciferase activity in the SPRY1-Wt group, while the luciferase activity in SPRY1-Wt group was not changed (Figure 3(b)). Overall, miR-21 could directly target SPRY1.

### 3.4. miR-21 Inhibited SPRY1 Expression and Facilitated CX43 Expression in VSMCs

As shown in Figure 4(a), the successful overexpression efficiency of miR-21 mimic was observed in T/G HA-VSMC cells. The mRNA and protein expression of SPRY1 were significantly reduced by miR-21 mimic in T/G HA-VSMC cells (Figures 4(b), 4(d), and 4(g)). On the contrary, miR-21 mimic dramatically augmented the mRNA and protein expression of CX43 (Figures 4(c), 4(e), and 4(g)). Moreover, there was no change before transfection. These results further proved that miR-21 targeted SPRY1 to modulate the expression of SPRY1.

### 3.5. miR-21 Accelerated Cell Multiplication and Inhibited Cell Apoptosis in VSMCs

Cell multiplication and apoptosis showed no evident differences between the two groups before transfection (Figures 5(a) and 5(d)). CCK-8 assay demonstrated that cell multiplication was facilitated by miR-21 mimic in T/G HA-VSMC cells (Figure 2(b)). Moreover, our data displayed that the apoptotic rate was lower in the miR-21 mimic group than that in the miR-NC group (Figures 5(c) and 5(e)). These results demonstrated that miR-21 played an oncogenic role in CHD progression.

## 4. Discussion

Accumulating evidence demonstrated that miRNAs acted as vital regulators in the progression of cardiovascular and cerebrovascular diseases, including CHD [25, 26]. For instance, miR-363 served as a modulator to generate the functional left-ventricular cardiomyocytes through negatively regulating HAND1 [27]. By targeting the NOR1/cyclin D pathway, miR-638 was revealed to participate in cell growth and metastasis of VSMCs [28]. A recent research reported that miR-23 was highly expressed in the plasma of patients with coronary artery disease, suggesting that miR-23 might be a novel biomarker for coronary artery disease [29]. It was reported that the miR-339 aggravated oxidative stress through regulating the Sirt2/Nrf2/FOXO3 axis, provided a potential therapy target for CHD [30]. By targeting IGF-1, miR-17 modulated the apoptosis and growth of human umbilical vascular endothelial cells in CHD [31]. Interestingly, miR-21 was reported to be upregulated in ischemic stroke [32]. Moreover, a previous study indicated that circulating miR-21 was related to the premature death risk in cardiovascular disease [33]. miR-21 was proved to be increased in peripheral blood mononuclear cells from CHD patients [34]. Consistent with these previous findings, our data showed that miR-21 was markedly upregulated in the plasma from patients with CHD compared with the controls. Besides, we also evaluated the functional role of miR-21 in CHD. Activation of endothelial cells and multiplication of VSMCs could induce the stenosis and occlusion of coronary artery wall, thereby aggravating the progression of CHD [35]. Thus, the effects of miR-21 on cell proliferation and apoptosis in VSMCs were explored in this study. Our results demonstrated that miR-21 dramatically boost cell proliferation and significantly repressed cell apoptosis in VSMCs. These findings indicated the promotion role of miR-21 in CHD progression.

SPRY1, a member of sprouty, was reported to be associated with the development of cardiovascular and cerebrovascular diseases. SPRY1 protein elevated collagen expression, thereby contributing to heart failure, arrhythmia, and even sudden cardiac death [36]. In addition, SPRY1 was lowly expressed in atherosclerosis mice and involved in the progression of atherosclerosis [37]. It was demonstrated that SPRY1 could effectively reduce VSMC multiplication in arteries [38]. In the current research, we found that SPRY1 was significantly downregulated in the plasma from CHD patients, suggesting that SPRY1 might be a crucial regulator in CHD progression. CX43 is a vital protein in the ventricle, and the abnormal increase of CX43 usually led to cardiac function impairment in patients [39]. Thus, we also measured the expression of CX43 in CHD patients and volunteers. Our results displayed that CX43 was markedly upregulated in the plasma from CHD patients, representing that CX43 played a regulatory role in CHD. Additionally, accumulating evidence proved that inflammatory cytokines might play vital roles in the progression of atherosclerosis [40]. In the present study, our data showed that the levels of the inflammatory cytokines including ICAM-1 and IL-1*β* were notably increased in the plasma from CHD patients, indicating that inflammation response was involved in the development of CHD.

TargetScan7.2 predicted that miR-21 harbored the potential binding sites with SPRY1. Previous studies noted that the target genes of miR-21 might be cell-specific, and SPRY1 was a target gene of miR-21 in cardiac fibroblasts, but not in cardiomyocytes [22]. In this research, dual-luciferase reporter assay verified that miR-21 directly targeted SPRY1 in VSMCs. Moreover, miR-21 could repress the expression of SPRY1 and enhance the expression of CX43 in VSMCs. Additionally, ICAM-1 or IL-1*β* level was positively correlated with miR-21 level in CHD patients. These findings suggested that miR-21 was involved in CHD progression through regulating SPRY1, CX43, and inflammation response. However, there were some limitations in this study. More plasma samples should be collected from CHD patients and volunteers for analysis, and other cell lines of coronary arteries and heart need to be used to explore the functional role of miR-21 in CHD progression. Moreover, the detailed mechanism among miR-21, SPRY1, and CX43 will be investigated in future study.

## 5. Conclusion

To sum up, increased miR-21, CX43, and inflammatory cytokines including ICAM-1 and IL-1*β*, as well as decreased SPRY1 in CHD patients, played important roles in CHD progression. Moreover, miR-21 could effectively promote cell multiplication and inhibit cell apoptosis in VSMCs via inhibiting SPRY1, providing a potential therapy target for CHD.

## Figures and Tables

**Figure 1:** Plasma levels of miR-21, SPRY1, and CX43. (a) The relative expression level of miR-21 in the plasma from CHD patients and healthy volunteers was detected using RT-qPCR analysis. (b) The mRNA expression of SPRY1 in the plasma from CHD patients and healthy volunteers was measured using RT-qPCR analysis. (c) The mRNA expression of CX43 in the plasma from CHD patients and healthy volunteers was determined using RT-qPCR analysis. (d, f) Western blot was used to assess the protein expression of SPRY1 protein in the plasma from CHD patients and healthy volunteers. (e, f) Western blot was used to examine the protein expression of CX43 in the plasma from CHD patients and healthy volunteers. (f) The representative images from western blot results. ^∗^*P* < 0.05.

**Figure 2:** Plasma levels of inflammatory cytokines. (a) The level of ICAM-1 in the plasma from CHD patients and healthy volunteers was detected using ELISA. (b) The level of IL-1*β* in the plasma from CHD patients and healthy volunteers was measured using ELISA. (c) Pearson analysis displayed that ICAM-1 was positively correlated with miR-21. (d) Pearson analysis showed that IL-1*β* was positively correlated with miR-21. ^∗^*P* < 0.05.

**Figure 3:** Targeting relationship between miR-21 and SPRY1. (a) miR-21 has the binding sites with SPRY1. (b) The luciferase activity in T/G HA-VSMC cells cotransfected with SPRY1-Wt, SPRY1-Mut, miR-21 mimic, and miR-NC was evaluated using dual-luciferase reporter assay. ^∗^*P* < 0.05.

**Figure 4:** Levels of miR-21, SPRY1, and CX43 in cells. (a) The relative expression of miR-21 was assessed by RT-qPCR analysis. (b) The relative mRNA expression of SPRY1 was determined by RT-qPCR analysis. (c) RT-qPCR analysis was utilized for CX43 mRNA expression measurement. (d, g) Western blot was performed to detect SPRY1 protein expression. (e, g) CX43 protein expression was determined by western blot. (f) The representative images from western blot results. ^∗^*P* < 0.05.

**Figure 5:** The effects of miR-21 on cell multiplication and apoptosis of T/G HA-VSMC cells. (a, b) Cell multiplication was evaluated by CCK-8 assay. (c–e) Cell apoptosis was determined using flow cytometry. ^∗^*P* < 0.05 vs. miR-NC; ^#^*P* < 0.05 vs. 24 h and ^∗^*P* < 0.05 vs. 48 h.

**Table 1:** Related primers.

	Upstream primer	Downstream primer
SPRY1	5′-GCAGTTCGTTAGTTGTGAT-3′	5′-GCAGTAGGCTGAATCTCT-3′
CX43	5′-TCTCGCCTATGTCTCCTCCTGG-3′	5′-AGTTAGAGATGGTGCTTCCCGC-3′
miR-21	5′-GCCCATCCTCAAATACAAAGC-3′	5′-GGTCCYGAACACAAAATGAGC-3′
*β*-Actin	5′-CCGTTCCGAAAGTTGCCTTTT-3′	5′-ATCATCCATGGTGAGCTGGC-3′
U6	5′-ATTGGAACGATACAGAGAAGATT-3′	5′-GGAACGCTTCACGAATTTG-3′

## Data Availability

The labeled dataset used to support the findings of this study are available from the corresponding author upon request.

## Additional Points

*Highlights*. (1) miR-21 was highly expressed in CHD. (2) miR-21 targeted SPRY1 in VSMCs. (3) miR-21 promoted CHD progression via targeting SPRY1.
